This article has been retracted.

# Thioredoxin Glutathione Reductase as a Novel Drug Target: Evidence from *Schistosoma japonicum*

**DOI:** 10.1371/journal.pone.0031456

**Published:** 2012-02-22

**Authors:** LiJun Song, JiaHuang Li, ShuYing Xie, ChunYan Qian, Jie Wang, Wei Zhang, XuRen Yin, ZiChun Hua, ChuanXin Yu

**Affiliations:** 1 Key Laboratory on Technology for Parasitic Disease Prevention and Control, Ministry of Health, Jiangsu Institute of Parasitic Diseases, Wuxi, Jiangsu, People's Republic of China; 2 The State Key Laboratory of Pharmaceutical Biotechnology, Nanjing University, Nanjing, Jiangsu, People's Republic of China; 3 Department of Schistosomiasis Diagnosis, Jiangxi Institute of Parasitic Disease, Nanchang, Jiangxi, People's Republic of China; Stanford, United States of America

## Abstract

**Background:**

Schistosomiasis remains a major public health concern affecting billions of people around the world. Currently, praziquantel is the only drug of choice for treatment of human schistosomiasis. The emergence of drug resistance to praziquantel in schistosomes makes the development of novel drugs an urgent task. Thioredoxin glutathione reductase (TGR) enzymes in *Schistosoma mansoni* and some other platyhelminths have been identified as alternative targets. The present study was designed to confirm the existense and the potential value of TGR as a target for development of novel antischistosomal agents in *Schistosoma japonicum*, a platyhelminth endemic in Asia.

**Methods and Findings:**

After cloning the *S. japonicum* TGR (SjTGR) gene, the recombinant SjTGR selenoprotein was purified and characterized in enzymatic assays as a multifunctional enzyme with thioredoxin reductase (TrxR), glutathione reductase (GR) and glutaredoxin (Grx) activities. Immunological and bioinformatic analyses confirmed that instead of having separate TrxR and GR proteins in mammalian, *S. japonicum* only encodes TGR, which performs the functions of both enzymes and plays a critical role in maintaining the redox balance in this parasite. These results were in good agreement with previous findings in *Schistosoma mansoni* and some other platyhelminths. Auranofin, a known inhibitor against TGR, caused fatal toxicity in *S. japonicum* adult worms in vitro and reduced worm and egg burdens in *S. japonicum* infected mice.

**Conclusions:**

Collectively, our study confirms that a multifunctional enzyme SjTGR selenoprotein, instead of separate TrxR and GR enzymes, exists in *S. japonicum*. Furthermore, TGR may be a potential target for development of novel agents against schistosomes. This assumption is strengthened by our demonstration that the SjTGR is an essential enzyme for maintaining the thiol-disulfide redox homeostasis of *S. japonicum*.

## Introduction

Schistosomiasis is a major tropical disease endemic in Africa, South America and Asia. It is estimated that approximately 600 million people are infected with the causative parasites in 76 countries around the world, and the disease results in about 20 million deaths annually [1]–[3]. In China, this disease caused by *Schistosoma Japonicum* remains a major public health concern, with more than 30 million people infected [4]. Currently, the control of schistosomiasis mainly depends on drug-based chemotherapy [5]. Since praziquantel was developed in the 1980s, it has replaced other drugs and became the first treatment of choice for schistosomiasis [6], [7]. However, praziquantel resistance or tolerance may arise after long-term, repeated large-scale chemotherapy is implemented. Decreased sensitivity of *Schistosoma mansoni* to praziquantel has been found in some endemic areas [8]–[12], and several case reports of failure of repeated standard praziquantel treatment to clear *Schistosoma haematobium* infections have also been reported [13], [14]. Although reduced sensitivity of *S. japonicum* to praziquantel has not been proven to date, the efficacy of the drug was reported to vary in different strains of this species [15]. Therefore, developing new antischistosomal agents to curb the emergence of drug-resistant schisotomes should be given a high priority.

Organisms are continuously attacked by endogenous and exogenous reactive oxygen species (ROS). Affluent antioxidant defense systems maintain the balance of pro-oxidants and anti-oxidants in a stable redox state and protect the homeostasis of the body. Two major systems exist to detoxify ROS in eukaryotes, the thioredoxin (Trx) system and the glutathione (GSH) system [16]. The Trx system is composed of nicotinamide-adenine dinucleotide phosphate (NADPH), Trx reductase (TrxR) and Trx. The GSH system consists of NADPH, GSH reductase (GR) and GSH. GR drives a tripeptide GSH-dependent system. Meanwhile, TrxR is an NADPH-dependent selenoprotein containing the thiol-disulfide redox active center [17], a GCUG active site motif located at the carboxyl terminus where “U” represents selenocysteine. As an important element in the active center of selenoproteins [18], [19], selenocysteine is exposed on the highly extended C-terminal surface of TrxR. The Cys and SeCys residues in the reduced state have strong pro-nuclear properties. Many electrophilic compounds can selectively and irreversibly combine with the active center [20], [21]. Both the Trx and GSH redox systems play an important role in the anti-oxidative network, regulation of transcriptional factors, cell growth and differentiation, synthesis of DNA, hormone action, cytokine function and metabolism of selenoproteins. At present, TrxR is considered a potential target for the development of novel drugs against tumors and infectious pathogens [20], [21].

In contrast to their mammalian hosts, thiol-disulfide redox homeostasis in platyhelminths such as *S. mansoni* [22], larval *Taenia crassiceps* (cysticerci) [23] *Echinococcus granulosus* [24] and *Fasciola hepatica* [25], fully depend on thioredoxin glutathione redutase (TGR) of linked thioredoxin-glutathione systems. It has been demonstrated that there are no separate TrxR and GR enzymes in *S. mansoni* and other platyhelminths. The functions are replaced by the unique multi-functional enzyme―TGR. *S. mansoni* TGR (SmTGR) with the activities of TrxR, GR and glutaredoxin (Grx) has been confirmed by RNA interference as an essential enzyme for *S. mansoni* survival [26]. Like all eukaryotic TrxR isoforms, TGR is a selenoprotein with a GCUG active motif at the carboxyl terminus [27]. Selenocysteine (U) is recoded by a dedicated UGA codon in the selenoprotein mRNA by translation machinery utilizing a specialized structural element, the selenocysteine insertion sequence (SECIS). Following the silencing of TGR expression or inhibition of its activity in *S. mansoni*, the parasites die of oxidative damage from the host, suggesting that SmTGR would be a promising and potential drug target [28].

In this study the components involved in maintaining redox balance in *S. japonicum* were investigated through a bioinformatic approach. Several expressed sequence tags (ESTs) homologous to the SmTGR gene, but no separate TrxR or GR gene, were found implying that the TGR gene may also exist in *S. japonicum* and plays an important role in redox balance. However, no information on the *S. japonicum* TGR (SjTGR) enzymatic system is currently available. Here we report the gene cloning, protein expression and purification, as well as enzyme characterization of SjTGR. The effect of auranofin, a known inhibitor of TGR [23], [24], [26], [29], against SjTGR was also assessed. The experimental findings further support TGR as a potential target for development of novel drugs against schistosomiasis.

## Methods

### Ethical statement

The animal work was approved by the Institutional Review Board (IRB00004221) of Jiangsu Institute of Parasitic Diseases, Wuxi, China (Permit Number: JIPDAERP20100724). All animals used in this work were conventionally housed in facilities and were provided food and water *ad libitum*. Animal studies including infection, intraperitoneal injection, orbital venous bleeding of mice were conducted in accordance with the recommendations in the Guidelines for the Care and Use of Laboratory Animals of the Ministry of Science and Technology of People's Republic of China ([2006]398). Mice were sacrificed by carbon dioxide asphyxiation in sealed containers according to the Guidelines. All efforts were made to minimize suffering.

### Reagents

5, 9-dithiobis (2-nitrobenzoic acid) (DTNB), glutathione disulfide (GSSG) and GSH were purchased from BIO BASIC INC (Toronto, Canada). The reduced form of NADPH was purchased from Roche (Basel, Switzerland), and RPMI 1640 was from Gibco (Invitrogen Corporation, Carlsbad, CA, USA). β-hydroxyethyl isulfide (HED), insulin and yeast GR was obtained from Sigma (St. Louis, MO, USA). Auranofin was purchased from ALEXIS (Lausen, Switzerland). The pGEM-T TA vector was from Promega (Madison, WI, USA). Finnzymes' Phusion® high fidelity polymerase was purchased from New England Biolabs (Ipswich, MA, USA). Recombinant Trx of *S. japonicum* was prepared in our lab. Illustra QuickPrep™ mRNA purification kit came from GE Healthcare Life Sciences (Piscataway, NJ, USA). SuperScript™ III First Strand Synthesis System was purchased from Invitrogen. The plasmids pET41a (+) and pSUABC were kindly provided by Elias S. J. Arnér (Department of Medical Biochemistry and Biophysics, Karolinska Institute, Stockholm, Sweden).

### Parasites and animals

*S. japonicum* cercariae (strain isolated in Jiangsu, China), hatched from infected *Oncomelania hupensis*, were provided by the Department of Snail Biology, Jiangsu Institute of Parasitic Diseases. Mice (C57BL/6), weighing 22∼24 g, were purchased from the Shanghai Sub-Center of Experimental Animals, Chinese Academy of Sciences, and raised in the Department of Experimental Animals, Jiangsu Institute of Parasitic Diseases.

### Preparation of mRNA and first strand cDNA of *S. japonicum* adult worms

Each mouse was infected with 50 *S. japonicum* cercariae by abdominal skin penetration. All mice were sacrificed on day 45 post-infection, and *S. japonicum* adult worms were collected through portal vein perfusion [30]. The mRNA from 0.5 g of *S. japonicum* adult worms was prepared by using the Illustra QuickPrep™ mRNA purification kit following the manufacturer's procedures. The first strand cDNAs were synthesized using mRNA of *S. japonicum* adult worms using the SuperScript™ III First Strand Synthesis System in accordance with the manual's instructions.

### Cloning of *S. japonicum* TGR gene

The ESTs of TGR in *S. japonicum* were BLAST searched with the *S. mansoni* TGR DNA sequence. The potential open reading frame of SjTGR was deduced by comparing all SjTGR ESTs to the DNA sequence of SmTGR. A pair of gene specific primers were designed according to the DNA sequence of the deduced open reading frame of SjTGR, and the primer sequences were as follows: forward primer: 5′-AACATATGCCTCCGATTGATGGAACA-3′ and reverse primer 1: 5′-TC AGCAACCGGTTACCGCTGCAGAGCCCCCA-3′.

The first strand cDNA of *S. japonicum* adult worms was used as the template to amplify the open reading frame DNA fragment encoding SjTGR using a high fidelity DNA polymerase. The specific DNA fragment was cloned into the pGEM-T vector after attaching a deoxyadenine at the 3′ terminal by Taq DNA polymerase and confirmed by sequencing at Invitrogen Corporation.

### Construction of the recombinant SjTGR expression plasmid

The chimeric gene composed of the SjTGR open reading frame plus a typical bacterial SECIS element was prepared by overlapping PCR using the following primer pair: forward primer: 5′-AACATATGCCTCCGATTGATGGAACA-3′ and reverse primer 2: 5′-GTCGACGGGCGCATAGGTTAACGATTGGTGCAGACCTGCAACCGATTATTAACCTCAGCAACCGGTTACCGC-3′. The reverse primer 2 included the bacterial SECIS: 5′-GGTTAATCGGTTGCAGGTCTGCACCAATCGTTAACCTATGCGCCC-3′ [31]. The 5′ *Nde* I site and 3′ *Sal* I site were introduced into the chimeric gene by PCR for cloning into the plasmid pET41a containing the corresponding restriction sites. The insertion in the resulting recombinant expression plasmid SjTGR-pET41a was confirmed by DNA sequencing at Invitrogen Corporation.

### Expression and purification of recombinant SjTGR

The recombinant SjTGR-pET41a vector and pSUABC vector, which expresses *sel*A, *sel*B and *sel*C to assist selenocysteine incorporation into the selenoprotein, were co-transformed into *Escherichia coli* BL21 (DE3) competent cells as described by Kuntz and colleagues [26]. The bacteria grown on Luria–Bertani (LB) medium plates containing ampicillin (100 µg/mL) and chloramphenicol (30 µg/mL) antibiotics were selected as positive clones. Single colonies containing the SjTGR-pET41a and pSUABC plasmids were incubated in LB medium containing L-cysteine and seleniate. When the absorbance value of the bacteria culture at 600 nm reached 2.4, IPTG was added at a final concentration of 0.5 mM. The bacteria were then grown at 24°C for 24 h to induce SjTGR expression. The expression products were analyzed on a 12% SDS-PAGE gel stained with Commassie Blue.

To confirm that the recombinant SjTGR was a selenoprotein, the bacteria containing the SjTGR-pET41a and pSUABC plasmids or those containing only the SjTGR-pET41a plasmid were inoculated into LB culture medium or induced in LB medium containing isotope ^75^Se-cysteine (SeCys). SeCys incorporation was analyzed on SDS-PAGE gels and autoradiograms.

The recombinant SjTGR was purified by affinity chromatography with an adenosine -2′,5′-diphosphate agarose (ADP-agarose, Sigma) [32]–[34]. Briefly, the bacteria cultures were collected by centrifugation, and the pellets were frozen and thawed repeatedly until they became transparent. Deoxyribonuclease was added to the bacteria lysates to digest the DNA. The lysate solutions were then centrifuged at 30,000× *g* for 30 min at 4°C, and the supernatants were passed through 0.45 µm filters. Samples in all steps above were kept on ice.

ADP-agarose column was equilibrated with buffer containing 50 mM potassium phosphate and 3 mM EDTA, pH 7.5. Supernatants containing the expressed products above were diluted ten-fold with the equilibration buffer, applied to the column, which was rinsed with wash buffer (0.4 M potassium phosphate, 3 mM EDTA, pH 7.5) until the ultraviolet absorption of the effluent did not decline further. The recombinant SjTGR proteins were then eluted with buffer containing 50 mM potassium phosphate and 0.5 M KCl, pH 7.5, and the fractions were analyzed by SDS-PAGE. The fractions containing SjTGR were pooled and applied to another ADP-agarose column, and the recombinant SjTGR proteins were eluted specifically with an NADPH linear gradient (0–0.5 mM) in 50 mM phosphate (pH 7.5). The fractions containing purified SjTGR proteins were pooled again and stored at −70°C after being dialyzed and concentrated by ultrafiltration (Amicon Ultra, Millipore, Bedford, MA, USA).

### Production of antiserum against recombinant SjTGR and immunoblotting

The purified recombinant SjTGR proteins were mixed with Freund's complete adjuvant (Sigma) to form water in oil emulsions. Each mouse was immunized intradermally in the cervical and back skin with 100 µL of the adjuvanted antigen (containing 50 µg recombinant SjTGR) and boosted two times with the same amount of Freund's incomplete adjuvant antigen at two week intervals. Blood samples were collected via the orbital vein on day 7 after the second boost. Antibody titers of sera against recombinant SjTGR were measured by conventional ELISA.

Purified recombinant SjTGR proteins and the *S. japonicum* adult worms homogenates were separated on SDS-PAGE gel and transferred to nitrocellulose (NC) membrane. After blocking with 5% milk powder solution for 1 h at room temperature, the NC membrane was incubated with the SjTGR antiserum diluted 1∶100 in PBST (PBS with 0.05% Tween-20) for 2 h at room temperature. The membrane was washed 3 times with PBST, for 10 min each time, and then incubated with HRP-conjugated goat anti-mice IgG (1∶3000 dilution, Bethyl) at room temperature for 2 h. After washing 3 times as above, the colored signals on the membrane were developed with DAB substrate (6 mg 3,3′-Dianinobenzidine dissolved in 10 ml PBS, 20 µl H_2_O_2_).

### SjTGR enzymatic assays

TrxR, GR and Grx activities of recombinant TGR were analyzed based on the methods described by Kuntz *et al.* [26] with a UV-visible spectrophotometer (UV-2550, SHIMADZU) at 25°C. The TrxR activity was determined by the 5, 5′-diothiobis (2-nitrobenzoic acid) (DTNB) reduction assay and the insulin reduction assay. The DTNB reduction assay solution contained 100 µM NADPH, 3 mM DTNB, 10 mM EDTA in 0.1 M potassium phosphate (pH 7.4). The increase of absorbance at 412 nm was monitored during the first 2 min. The extinction coefficient of 13.6 mM^−1^ cm^−1^ for TNB was used in the calculation. One enzyme unit is defined as the NADPH-dependent production of 2 µmol of 2-nitro-5-thiobenzoic acid per min at 25°C.

Trx reduction assay was determined by monitoring the decrease of NADPH consumption at 340 nm during the first 2 min. The assay was carried out in the presence of 1 mg/ml insulin, 10 µM SjTrx and 100 µM NADPH in 0.1 M potassium phosphate (pH 7.4) containing 10 mM EDTA. The extinction coefficient of 6.22 mM^−1^ cm^−1^ for NADPH was used in the calculation. One unit of TrxR activity is defined as the oxidation of 1 µmol of NADPH per min at 25°C.

The GR activity was determined with GSSG. The reaction mixture contained 100 µM NADPH, 100 µM GSSG in 0.1 M potassium phosphate (pH 7.4) containing 10 mM EDTA. Decrease of NADPH consumption at 340 nm during the first 2 min was monitored. The extinction coefficient of 6.22 mM^−1^ cm^−1^ for NADPH was used in the calculation. One unit GR activity is defined as the oxidation of 1 µmol of NADPH per min at 25°C.

The Grx activity was determined by monitoring decrease of NADPH consumption at 340 nm during the first 2 min, and the assay was performed in the presence of 1 mM GSH, 8 mM HED, 0.6 units of yeast GR, 100 µM NADPH in 0.1 M potassium phosphate (pH 7.4) containing 10 mM EDTA. The extinction coeffcient of 6.22 mM^−1^ cm^−1^ for NADPH was used in the calculation. One unit of Grx activity is defined as the oxidation of 1 µmol of NADPH per min at 25°C. All assays were performed in triplicate.

### Kinetic analysis

Based on the method described by Kuntz *et al.* [26], SjTGR activities with NADPH, DTNB, SjTrx, GSSG, HED and GSH were determined in the following buffer: 100 µM NADPH, 10 mM EDTA, 0.1 M potassium phosphate (pH 7.4) and 48 nM SjTGR. In the TrxR activity assay, DTNB concentrations varied from 100 to 1000 µM, NADPH concentrations from 5 to 100 µM and Trx concentrations from 9 to 34 µM. In the GR activity, GSSG concentrations were from 10 to 100 µM, and NADPH was from 5 to 100 µM. In the Grx assay, 2 to 10 mM HED, 100 to 1500 µM GSH and 10 to 100 µM NADPH were used. In each reaction, the concentration of one substrate was changed while keeping the others constant. Kinetic parameters were obtained by curve fitting of experimental data using OriginPro 7.0. All assays were performed in triplicate.

### Auranofin inhibition of recombinant SjTGR

Inhibition of TrxR, GR and Grx activities of recombinant SjTGR by different concentrations of auranofin was determined in the enzyme assays described above. The 50% inhibitory concentration (IC_50_) values of auranofin in the various assays were calculated by curve fitting using the SPSS 13.0 statistical software.

The inhibitory constants () of auranofin for TrxR activity and GR activity of SjTGR were assessed using varying substrate and inhibitor concentrations as follows: DTNB 100, 150, 200, 300, 500, 700, 1000 µM; GSSG 10, 15, 20, 30, 50, 70, 100 µM; auranofin 5, 10, 20, 30 nM. The  values were calculated using the following equations [35]:(1)
(2)Formula (1) is used for calculating  of competitive inhibition. Where  is the apparent  at different inhibitor concentrations, and  is the inhibitor concentration.

Formula (2) is used for calculating of non-competitive inhibition. Where is the apparent  at different inhibitor concentrations, and  is the inhibitor concentration.

All assays were performed in triplicate.

### Toxicity of auranofin on *S. japonicum* adult worms in vitro

Stock solutions of auranofin and praziquantel were prepared by dissolving 1 mg of the drugs in 0.4 ml dimethyl sulfoxide (DMSO) and adding 0.6 ml RPMI 1640 medium. *S. japonicum* worms obtained from mice (C57BL/6, male, 22∼24 g, each infected with 50 cercariae) were washed in RPMI 1640 medium, kept at pH 7.5 with HEPES 20 mM and supplemented with penicillin (100 UI·mL^−1^), streptomycin (100 µg·mL^−1^) and 10% bovine fetal serum (Gibco) [36]. After washing, two pairs of adult worms were transferred to each well of a 24-well culture plate containing 2 mL of the same medium. The worms were cultured for 30 to 60 min at 37°C in a humid atmosphere containing 5% CO_2_, and then different concentrations of auranofin (1, 5, 10, 20 and 30 µg/ml) diluted with RPMI 1640 medium were added. Control worms were treated with equal volumes of RPMI 1640 or DMSO, and worms treated with 30 µg/mL praziquantel were also observed. The worm mobility, tegumental alterations and parasite survival were monitored under an inverted microscope (Leica, Germany) at 1, 6, 24, 48 and 72 h. Parasite death was defined as having no motor activity during 2 min of continuous observation as well as morphological and tegumental alterations [37]. Worms treated with auranofin were homogenized in 0.1 M potassium phosphate (pH 7.4). The homogenates were centrifuged at 20,000× *g* for 1 h at 4°C, and the supernatants were assayed for TrxR and GR activities as described above. All assays were repeated three times.

### Auranofin treatments in vivo

A stock solution of auranofin was prepared by dissolving 2 mg of the drug in 0.4 mL DMSO and adding 0.6 mL of aseptic 0.9% sodium chloride. The stock solution was diluted to 0.4 mg/mL with the aseptic 0.9% sodium chloride before use. All mice (C57BL/6, male, 22∼24 g) infected with 30 *S. japonicum* cercariae by abdomenal skin exposure were administered 6 mg/kg auranofin injected intraperitoneally twice daily for 5 days beginning 35 days post-infection. Control mice were given the same dose of carrier on the same timetable. Mice were sacrificed on day 42 post-infection. Worms were counted by portal vein perfusion. Liver tissues were digested with 5% potassium hydroxyl solution, and the eggs from the liver tissue were counted. The worm reduction rate and egg reduction rate were calculated using the following formulas.

Worm reduction rate (%)(mean number of adult worms per mouse in control group - mean number of adult worms per mouse in experimental group)mean number of adult worms in control group.

Egg reduction rate (%)(mean number of eggs per mouse in control group - mean number of eggs per mouse in experimental group)mean number of eggs per mouse in control group.

### Statistical analysis

The numbers of worms and eggs per gram of liver were expressed as mean values ± standard errors (SD). Significant reductions in worm and egg burdens after auranofin treatment were determined by two-tailed Student *t*-test using statistical software SPSS 13.0. Differences between median values were considered to be significant at the level of 5%.

## Results

### Cloning and characterization of the SjTGR gene

The cDNA fragment encoding the open reading frame of the SjTGR protein was amplified from the mRNA of *S. japonicum* adult worms using a pair of gene specific primers designed according to the *S. japonicum* EST sequence, which showed a high degree of homology to the SmTGR gene. The cDNA fragment was composed of 1791 nucleotides encoding 598 amino acids. The predicted molecular weight of SjTGR was 64.9 kDa with an isoelectric point of 6.38. The amino acid sequence of SjTGR was 91% identical to SmTGR and 55% similar to human TrxR. Like SmTGR, the SjTGR protein contained NADPH- and FAD-binding domains, a dimer interface domain of pyridine nucleotide disulfide oxidoreductases and the thiol-dislifide redox active center (-CVNVGC-). A glutaradoxin active site (-CPFC-) was found in its N-terminus, and its C-terminus contained a conserved tetrapeptide sequence GCUG (U: selenocysteine), which is the catalytic domain of TGR [27].

### Expression and selenium incorporation of recombinant SjTGR

As the synthesis of selenoprotein depends on a highly species-specific translation mechanism, use of the bacterial-type SECIS element was necessary in order to express the SjTGR selenoprotein in *E. coli* host cells. The open reading frame DNA sequence of SjTGR was fused with the SECIS element by PCR to form a chimeric gene following the procedure described by Arnér and colleagues [31]. The chimeric SjTGR gene was cloned directionally into the expression plasmid pET41a at the restriction enzyme sites *Nde* I and *Sal* I, resulting in the recombinant plasmid SjTGR-pET41a. Restriction analysis and DNA sequencing confirmed that the chimeric SjTGR gene had been inserted into the pET41a expression plasmid correctly (Fig. 1).

**Figure 1:** Analysis of recombinant SjTGR-pET41a by enzyme restriction. (A) Agarose gel (1%) electrophoresis of recombinant SjTGR-pET41a or pET41a vectors. Lane 1: Purified PCR amplified SjTGR gene fragment of about 1,800 bp. Lane 2: Products of recombinant plasmid SjTGR-pET41a digested by *Nde* I/*Sal* I. The sizes of the pET41a backbone and the SjTGR gene were about 5,000 bp and 1,800 bp, respectively. Lane 3: Products of plasmid pET 41a digested by *Nde* I/*Sal* I. The sizes of the fragments from *Nde* I/*Sal* I digestion of pET41a were about 5,000 bp and 900 bp. Lane 4: Undigested pET 41a plasmid of 5933 bp. Lane 5: Undigested recombinant plasmid SjTGR-pET41a of about 6,800 bp. Note that both undigested plasmids migrated lower in the gel due to the super-helical structures. MW: DNA molecular weight marker. (B) Schematic diagram of the SjTGR-pET41a plasmid showing relevant enzyme sites and the SjTGR insert size.

The selenocysteine insertion during selenoprotein translation in *E. coli* requires an *E. coli*-type SECIS element just following the UGA codon in the selenoprotein mRNA, as well as the products of the *sel*A, *sel*B, and *sel*C and *sel*D genes [31]. In this study, the recombinant SjTGR-pET41a plasmid was co-transformed into *E. coli* BL21 with the pSUABC vector expressing the *sel*A, *sel*B and *sel*C genes (encoding selenocysteine synthase, SELB and tRNA^Sec^, respectively) to aid in the production of SjTGR as a putative selenoprotein. When the cells were induced with 1 mM IPTG for 4 h at 37°C, the SjTGR proteins were expressed in inclusion bodies, which appeared in the precipitate of the bacterial lysate obtained by ultrasonication. Little soluble recombinant SjTGR was found in the supernatant of the bacterial lysate (Fig. 2A). However, when the growth temperature was reduced to 24°C and the bacteria were induced with IPTG for 24 h beginning at the stationary growth stage (OD_600 nm_ of culture reaching 2.4) [38], soluble SjTGR proteins were produced successfully (Fig. 2B). The selenocysteine incorporation analysis using ^75^Se-labeling cysteine and autoradiograms showed that the products of *sel*A, *sel*B, and *sel*C could increase the yield of SjTGR, suggesting that it is a selenoprotein (Fig. 3).

**Figure 2:** Electrophoretic patterns of expression products of recombinant SjTGR. (A) Expression products from *E. coli* BL21 transformed with recombinant SjTGR-pET41a and induced with 1 mmole/L of IPTG at 37°C for 4 h. Lane 1: Supernatant of bacterial lysate. Lane 2: Precipitate of bacteria lysate resuspended with PBS. The black arrow indicates the expressed SjTGR protein band. MW: Protein molecular weight marker. (B) Expression products from transformed or non-transformed *E. coli* BL21 induced with 0.5 mmole/L of IPTG at 24°C for 24 h. Products in precipitates (lane 1) or supernatant (lane 2) of induced bacteria containing plasmid SjTGR-pET41a show expression of the recombinant SjTGR (black arrow). Expression products of induced bacteria containing plasmid pET41a (lane 3) or of induced non-transformed bacteria (lane 4) are also shown. MW: Protein molecular weight marker.

**Figure 3:** Analysis of isotope ^75^Se-cysteine incorporation. (A) Profile of expressed protein products on a 12% SDS-PAGE gel. (B) Autoradiogram profile of expressed products corresponding to the proteins on SDS-PAGE. Lane 1: Expression products of *E.coli* BL21 containing plasmid SjTGR-pET41a. Lane 2: Expression products of *E.coli* BL21 containing plasmids SjTGR-pET41a and pSUABC. MW: Protein molecular weight marker. The black dots on the SDS-PAGE gel are the expression products of *E.coli* BL21 containing plasmids SjTGR-pET41a and pSUABC. The expression products containing isotope ^75^Se-cysteine (SeCys) were dotted on the SDS-PAGE gel after electrophoresis as a positive control for autoradiography. The black arrow indicates the SjTGR selenoprotein developed by autoradiography.

The recombinant SjTGR protein was purified with an adenosine 2′, 5′-diphosphate agarose (Sigma A3515) column, used for specific affinity purification of NADPH-binding proteins. The purity of the SjTGR protein sample was more than 95% (Fig. 4), indicating the NADPH binding capacity of the recombinant SjTGR.

**Figure 4:** Protein profile of purified recombinant SjTGR. Lane 1: Purified recombinant SjTGR protein on SDS-PAGE gel stained with Commassie Blue. MW: Protein molecular weight marker.

### Western blotting with antiserum against SjTGR

High titer (>1∶204,800) antiserum against recombinant SjTGR was obtained after immunizing mice with the purified recombinant SjTGR. The antiserum could recognize a single protein band of expected size (MW ∼65 kDa) in the supernatant of *S. japonicum* adult worms homogenates by Western blotting (Fig. 5). The size of the recombinant SjTGR band was similar to that of the natural SjTGR. There were no other protein bands recognized by the antiserum. These results suggested that the recombinant SjTGR proteins were immunoreactive, inducing antibodies specific to the native SjTGR protein, and that no cross-reactive proteins were present in the *S. japonicum* adult worm.

**Figure 5:** Western blotting analysis of *S. japonicum* worm homogenate. Adult worm supernatant (lane 1) and purified recombinant SjTGR protein (lane 2) detected by mice polyclonal serum antibodies against recombinant SjTGR. MW: Protein molecular weight marker.

### Activity and kinetics of recombinant SjTGR

The enzyme activities of purified SjTGR were determined using a broad range of substrates, and the results showed that SjTGR possessed the characteristic activities of mammalian TrxR, GR and Grx. The specific activities were 8.11±0.34 µmol·min^−1^ mg^−1^ with DTNB, 3.33±0.08 µmol·min^−1^ mg^−1^ with Trx, 2.19±0.01 µmol·min^−1^ mg^−1^ with GSSG, and 12.10±0.39 µmol·min^−1^ mg^−1^ in a Grx assay coupled to HED. The TrxR activity (with substrates DTNB and Trx) and the Grx activity of SjTGR were similar to those of SmTGR, although the GR activity of SjTGR was lower than that of SmTGR (Table 1).

**Table 1:** Comparison of recombinant TGR enzyme activities of *S. japonicum* and *S. mansoni*.

Enzyme	Substrate	*S. japonicum* TGR (µmol·min^−1^ mg^−1^)	*S.mansoni* TGR [24] (µmol·min^−1^ mg^−1^)
TrxR	NADPH+DTNB	8.11±0.34	10.2
	NADPH+Trx	3.33±0.08	2.2
GR	NADPH+GSSG	2.19±0.01	7.2
Grx	NADPH+HED	12.10±0.39	9.9

The  of SjTGR with different substrates were 21.42±0.44 µM (NADPH), 3.24±0.40 µM (Trx), 145.05±6.31 µM (DTNB), 49.55±6.31 µM (GSSG), 2,792±231 µM (HED) and 3,831±54 µM (GSH) (Table 2), which were similar to those of SmTGR (Table 3). The catalytic efficiencies of SjTGR on TrxR, GR and Grx were different and found to be in the following order: TrxR (10^5^–10^6^ M^−1^·s^−1^)>GR (10^5^ M^−1^·s^−1^)>Grx (10^3^ M^−1^·s^−1^).

**Table 2:** Kinetics of recombinant SjTGR with different substrates.

Substrate	K*_m_* µM	V_max_ µM·min^−1^	K*_cat_* s^−1^	K*_cat_*/K*_m_* M^−1^·s^−1^
NADPH (DTNB)	21.42±0.44	31.45±0.83	10.92	5.10×10^5^
Trx	3.24±0.40	13.77±0.16	4.78	1.48×10^6^
DTNB	145.05±6.31	23.50±1.02	8.16	1.19×10^5^
NADPH (GSSG)	83.24±24.27	14.03±4.38	4.87	5.85×10^4^
GSSG	49.55±6.31	15.40±0.58	5.35	1.08×10^5^
NADPH (Grx)	10.97±2.42	43.01±0.18	14.93	1.36×10^6^
HED	2,792±231	24.92±0.67	8.65	3.10×10^3^
GSH	1,698±54	45.45±4.28	15.78	9.30×10^3^

Kinetic constants for recombinant SjTGR (48 nM) were determined in assays performed at 25°C in 0.1 M potassium phosphate (pH 7.4) with 10 mM EDTA and 100 µM NADPH. All assays were conducted in triplicate.

**Table 3:** Comparison of kinetics of recombinant TGR from *S. mansoni* and *S. japonicum* with different substrates.

Substrate	*S.mansoni* [26]			*S.japonicum*		
	K*_m_* µM	K*_cat_* s^−1^	K*_cat_*/K*_m_* M^−1^·s^−1^	K*_m_* µM	K*_cat_* s^−1^	K*_cat_*/K*_m_* M^−1^·s^−1^
NADPH	13.7	20.1	1.5×10^6^	21.42	10.92	5.10×10^5^
Trx	6.37	30	4.7×10^6^	3.24	4.78	1.48×10^6^
DTNB	114	16	1.4×10^5^	145.05	8.16	1.19×10^5^
GSSG	71.5	21.7	3.0×10^5^	49.55	5.35	1.08×10^5^
HED	1,867	17.8	9.6×10^3^	2,792	8.65	3.10×10^3^
GSH	248.6	20.1	8.1×10^4^	1,698	15.78	9.30×10^3^

Although the  values of recombinant SjTGR with various substrates were lower than those of SmTGR, the catalytic efficiencies () of both enzymes with the same substrate were similar (Table 3).

### Inhibition of recombinant SjTGR by auranofin

Inhibition of recombinant SjTGR by auranofin was observed by adding different amounts of the inhibitor into the enzyme assay system using DTNB, GSSG or HED as substrate. The experimental results showed that auranofin could inhibit the TrxR, GR and Grx activities of recombinant SjTGR, and the inhibitory effects were concentration dependent (Fig. 6A). The IC_50_ values were 6.89, 0.47 and 8.12 nM, respectively, for the DTNB, GSSG and HED substrates with 5 nM recombinant SjTGR. The inhibitory effect of auranofin on TrxR activity was competitive, increasing the  for substrates while the  remained constant. The inhibitory effect of auranofin on GR activity was non-competitive, altering the  while the  for substrates remained constant. The inhibitory constants () were 0.762 nm for TrxR activity and 0.034 nm for GR activity according to apparent  and  values with various concentrations of auranofin (Fig. 6B, 6C).

**Figure 6:** Inhibition of auranofin on enzymatic activities of recombinant SjTGR. (A) Percentages of TrxR, GR and Grx activities inhibited by different doses of auranofin with DTNB, GSSG or HED as substrate. (B) Inhibition constant () values of auranofin on recombinant SjTGR in the TrxR assay. The straight lines were fitted on the basis of the reciprocal of concentration of substrate and initial velocity. The concentrations of auranofin were 0 nM, 5 nM, 10 nM and 15 nM, and DTNB ranged from 60 to 1,000 µM. (C) Inhibition constant () values of auranofin on SjTGR in the GR activity assay. The straight lines were fitted on the basis of the reciprocal of concentration of substrate and initial velocity. The concentrations of auranofin were 0 nM, 5 nM, 10 nM and 20 nM, and GSSG ranged from 10 to 100 µM.

### Toxicity of auranofin in cultured *S. japonicum* adult worms

The effects of auranofin on cultured worm survival were observed by culturing the worms in medium containing different concentrations of auranofin, and the mobility and death rates of the parasites were monitored. Auranofin at 5 µg/ml (7.40 µM) resulted in a 53.3% decrease of worm viability after 6 h and 66.7% after 12 h. By 24 h, 100% mortality was observed. The median lethal dose (LD_50_) of auranofin was 2.56 µg/ml (3.78 µM) at 24 h, with 95% confidence interval 2.09∼3.02 µg/ml. Auranofin at 5 µg/ml (7.40 µM) reduced 57.1% of the TrxR activity and 71% of the GR activity in the *S. japonicum* adult worms homogenates compared to that of carrier treated-control worms, and the inhibitory effects were dose-dependent. No TrxR and GR activity was observed in the homogenates when the worms were treated with auranofin at 30 µg/ml (44.22 µM) (Fig. 7A). Additionally, the inhibitory effects of auranofin on TrxR and GR activities increased with time (Fig. 7B, 7C).

**Figure 7:** Inhibition of *S. japonicum* adult worms by auranofin in vitro. (A) Effects of auranofin (AUF 1, 5, 10, 20, 30 µg/ml) on TrxR and GR activities of adult worms after 3 h of treatment. Worms were mock treated in the control groups (RPMI 1640 and 1.2% DMSO). Worms were treated with 30 µg/ml of praziquantel in the PZQ 30 µg/ml group. (B) Inhibition of auranofin on TrxR activity of adult worms over time. Worms were treated with 5 and 10 µg/ml of auranofin, and the TrxR activities of worm homogenates were tested after 0, 1, 3 and 6 h. (C) Inhibition of auranofin on GR activity of adult worms over time. Worms were treated with 5 and 10 µg/ml of auranofin, and the GR activities of worm homogenates were tested after 0, 1, 3 and 6 h.

### In vivo activity of auranofin

ICR mice infected with 30 cercariae were treated with 6 mg/kg auranofin twice daily for 5 days beginning on day 35 post-infection. The results showed that auranofin could reduce worm burden by 41.50% and egg burden by 43.18% at the adult worm stage (Table 4).

**Table 4:** Treatment effect of auranofin on *S. japonicum* in mice.

Groups	Mice No.	Number of worms(Mean±SD)	Worm reduction rate (%)	Number Of Eggs per gram of liver (Mean±SD)	Egg reduction rate (%)
Control	11	23.25±5.91		96639.23±30692.60	
Auranofin	10	13.60±6.47	41.50*	54907.33±35530.09	43.18*

* Auranofin treatment versus control, *P*<0.01 by t-test.

## Discussion

The antioxidant system plays a critical role in physiological functions of an organism and protects schistosomes from host immune attack [16], [25]. Instead of having separate TrxR and GR enzymes, the single TGR protein in platyhelminths carrying these functions can completely deoxidize both Trx and GSSG [22]. TGR proteins of *S. mansoni* [22], larval *T. crassiceps* (cysticerci) [23], *E. granulosus* [24] and *F. hepatica* [25] have all been determined as potentially important drug targets. *S. mansoni* adult worms die when the activity of TGR is inhibited or silenced, as TGR produces partial or complete protective effects against oxidative damage in the host [26]. However, little attention has been focused on targeting the redox system of *S. japonicum*, a helminth endemic in Asia, for development of new schistosomicides.

In this study, the TGR gene of *S. japonicum* was cloned, and the deduced amino acid sequence of SjTGR revealed that it included NADPH- and FAD-binding domains, a thiol-disulfide redox active center (-CVNVGC-) and a Grx active site (-CPFC-). It was found to be 91% identical to SmTGR and 55% similar to human TrxR. There were 32 ESTs homologous to SmTGR found by analyzing ESTs of *S. japonicum.* One longer EST contained a conservative SECIS element in the non-translated region following the termination codon (TGA) of the TGR open reading frame. The SECIS element mediates the selenocysteine insertion at the penultimate amino acid of TGR functioning in concert with an adjacent cysteine as an essential part of this redox center [39], implying that SjTGR is also a selenoprotein enzyme like the mammalian TrxR isoforms. As selenoprotein synthesis is a highly species-specific process, we fused the SjTGR cDNA with the SECIS sequence of *E. coli* in constructing the recombinant SjTGR-pET41a plasmid in order to express the SjTGR selenoprotein in *E.coli* host cells [31]. Co-transformation of this plasmid into *E.coli* BL21 along with the pSUABC plasmid expressing *sel*A, *sel*B, and *sel*C that provided proteins to aid in the production of selenoproteins successfully yielded a soluble 65 kDa SjTGR protein upon IPTG induction. The selenocysteine incorporation analysis using ^75^Se-labeling cysteine and autoradiograms showed that the products of *sel*A, *sel*B, and *sel*C could increase the yield of SjTGR proteins. These results also confirmed that SjTGR is a selenoprotein.

Using the same methods previously published for production of recombinant SmTGR and conditions for enzyme kinetics analysis [26], the experimental data in the present study showed that SjTGR is a multifunctional enzyme with TrxR, GR and Grx activities. The GR activity of SjTGR was lower than that in SmTGR (2.19±0.01 µmol·min^−1^ mg^−1^ vs. 7.2 µmol·min^−1^ mg^−1^). However, the lower activity was compensated by the lower  value (Table 3). Comparison of the  values of SmTGR and SjTGR (3.0×10^5^ M^−1^·s^−1^ vs. 1.08×10^5^ M^−1^·s^−1^) indicated that the GR catalytic efficiencies of SjTGR and SmTGR were comparable.

The  with Trx (1.48×10^6^ M^−1^·s^−1^) was about 10 times that with GSSG (1.08×10^5^ M^−1^·s^−1^) and approximately 100 times that with HED (3.10×10^3^ M^−1^·s^−1^). These findings support the hypothesis that the catalytic efficiency of TGR with Trx was higher than that with GSSG and HED. The Trx/GSSG ratios of 3.3 and 15.7 in *T. crassiceps* [23] and *S. mansoni* [26] have also been reported. In all cases, TGR showed a preference toward Trx as substrate.

Compared to the TrxR  (21.42±0.44 µM) and GR  (83.24±24.27 µM) of SjTGR, the Grx  (10.97±2.42 µM) with NADPH was the lowest, which suggests that NADPH, combined with SjTGR, tends to deliver electrons to the Grx activity domain first and then to Trx. In *S. mansoni,* the electrons flow within the TGR domain from NADPH to the C terminus, then from the C terminus to either Trx or the Grx domain [40]. Electrons are selectively delivered to the acceptor by the C-terminal arm shuttling between SmTrx and the Grx domain [40]. Further study on the direction of electron transfer of SjTGR will be surveyed in our future work.

Compared to the typical human TrxR (2.2×10^6^ M^−1^·s^−1^) [41] and GR (3.2×10^6^ M^−1^·s^−1^) [42], it is obvious that the catalytic efficiencies of TrxR from helminths fall into the same range, but their GR catalytic efficiencies were all lower than that of human TrxR (Table 3). One possible reason for this phenomenon is that schistosomes may use the reduced GSH derived from host erythrocytes they ingest to maintain their redox balance, decreasing the requirement of GSSG reduction accordingly. Our results also provide evidence that schistosome TGR is not an efficient GR [40].

High titer (>1∶204,800) antiserum was obtained after immunizing mice with the purified recombinant SjTGR. In Western blot analysis, the polyclonal antibodies in this antiserum could recognize a ∼65 kDa protein band corresponding to the expected size of SjTGR in the supernatant of *S. japonicum* adult worms homogenates, indicating that the recombinant SjTGR was immunogenic and induced antibodies reactive to the natural protein. Furthermore, this antiserum did not react with other bands in the worm supernatant. Since the amino acid sequence of TGR is highly homologous to the 56 kDa TrxR and 52 kDa GR of eukaryotic cells, if individual TrxR or GR proteins exist in the *S. japonicum* adult worm, the corresponding cross-reactive protein bands would have been detected. These results indicate that the *S. japonicum* adult worm does not express separate TrxR or GR molecules, the functions of which are entirely replaced by TGR. This point was also confirmed by bioinformatic analysis which found no TrxR or GR EST sequences in the *S. japonicum* EST database (data not published). These data reported here suggest that SjTGR plays a key role in the maintenance of redox balance in *S. japonicum*.

In the study, the gold compound auranofin, a known inhibitor of TGR, was found to inhibit the activity of the recombinant SjTGR. The IC_50_ values of auranofin against TrxR, GR and Grx activities were in the nanomolar range (6.89, 0.47, 8.12 nM) with 5 nM recombinant SjTGR. Of note, the IC_50_ value of auranonfin on GR in *S. mansoni* worms was almost 9 times higher than that in *S. japonicum,* while the IC_50_ values against TrxR and Grx were nearly the same. Interestingly, the inhibitory mechanisms of auranofin against TrxR and GR were distinct. Auranofin-mediated inhibition of TrxR activity was competitive, while that of GR activity was non-competitive. This may be due to differences in the structures of auranofin, DTNB and GSSG. Auranofin has a benzene ring structure [43], which is similar to DTNB with two benzene rings connected by a disulfide bond [44], but different from the carbon chain of GSSG [45]. Auranofin and DTNB may combine with the active center of TGR competitively, but auranofin may combine outside of the active center of GR to influence the GR activity of SjTGR in a non-competitive manner. The  value of auranofin on TrxR and GR was very low (0.762 nM and 0.034 nM), indicating that just a small amount of auranofin could completely inhibit SjTGR activity, similar to the findings in *larval T. crassiceps* [23], *E. granulosus* [24] and *S. mansoni* [43].

Auranofin was confirmed to be toxic to *S. japonicum* adult worms *in vitro*, and the dose of 5 µg/ml (7.40 µM) resulted in 100% mortality after 24 h. The calculated LD_50_ of auranofin against *S. japonicum* adult worms *in vitro* was 2.56 µg/ml (3.78 µM) at 24 h. These results are in agreement with those reported from *S. mansoni* adult worms [26], *E. granulosus* larval worms [46] and *T. crassiceps* metacestode [47]. *In vivo,* 6 mg/kg auranfin could partially cure *S. japonicum*-infected mice, with a 41.50% reduction in worm burden and a 43.18% reduction in egg burden. We obtained similar results to those previously observed in *S. mansoni* treated with auranofin [26].

As SjTGR is highly similar to SmTGR in terms of amino acid sequence and activities, it may be a potentially important drug target as well. However, there are some differences between SmTGR and SjTGR. The Grx activity motif of SjTGR is composed of CPFC compared to CPYC in SmTGR [27]. The differences in amino acid sequence in the TrxR domain of TGR between *S. mansoni* and *S. japonicum* are more marked [39]. The potential differences in the molecular structures between SjTGR and SmTGR may result in different inhibitory effects of drugs targeting these proteins. Of course, further protein homology modeling and crystallographic structural studies will be required to better understand TGR as a drug target. Such studies can benefit in the development of new chemotherapeutic drugs targeting multiple schistosome species. Meanwhile, the unique aspects of the SjTGR structure may help to improve potency of these new drugs against *S. japonicum.*

In conclusion, our study confirms that a multifunctional enzyme SjTGR selenoprotein, instead of separate TrxR and GR enzymes, exists in *S. japonicum*, which is an extension of findings on TGR in other platyhelminths. SjTGR plays an essential role in maintaining the redox balance in *S. japonicum,* which further confirms TGR as a potential target for the development of new drugs against schistosomiasis.
